# Analysis of Multiple Vitamins Serum Levels and Disease-Related Factors in Children with Acute Leukemia

**DOI:** 10.1155/2022/5330563

**Published:** 2022-04-15

**Authors:** Zeliang Song, Juanjuan Li, Jing Cao, Lei Zhang, Zhaoxia Zhang, Shunqiao Feng, Dixiao Zhong, Mei Yue, Mengze Hu, Rong Liu

**Affiliations:** Department of Pediatric Hematology Oncology, Children's Hospital, Capital Institute of Pediatrics, No. 2, YaBao Road, Chaoyang District, Beijing 100020, China

## Abstract

**Objective:**

To explore the relationship between vitamins levels and disease-related indicators in children with acute leukemia (AL).

**Methods:**

A total of 107 hospitalized children with AL were enrolled in this study and assigned to one group in each of the following categories: infected group (*n* = 52) and noninfected group (*n* = 55); treatment remission group (*n* = 56) and nonremission group (*n* = 51); high-risk (HR) group (*n* = 44), intermediate risk (IR) group (*n* = 53), and slight risk (SR) group (*n* = 8); cyclophosphamide + cytosine arabinoside+6-mercaptopurine + pegaspargase group (CAML, *n* = 15); methotrexate group (MTX, *n* = 9); and vindesine + daunomycin + L-asparaginasum + prednisone (VALP, *n* = 38). Hematological and serological parameters, hepatic and renal function, and changes in vitamins A, B1, B2, B6, B9, B12, C, D, and E serum content in children with AL were analyzed to investigate their relationship with AL disease-related factors.

**Results:**

The vitamin D level was significantly higher in the noninfected group than in the infected group (*P* < 0.05). Compared with the nonremission group, the level of vitamin B1 in the treatment remission group was significantly higher, while the levels of vitamin B6 and B12 were notably lower (*P* < 0.05). The levels of vitamins B6 and B12 were notably different among the treatment groups. Multivariate analysis showed that hemoglobin (Hb) and C-reactive protein (CRP) were predisposing factors of AL in children. The disease type (acute lymphoblastic leukemia/acute myelogenous leukemia) was the factor affecting remission in AL children. Abnormal kidney function and the occurrence of icterus were the influencing factors for the risk degree in AL children. Platelet (PLT) count, activated partial thromboplastin time (APTT), neutrophils (N), and immunophenotype were shown to affect the choice of therapeutic regimens.

**Conclusion:**

There are notable vitamins imbalances in children with AL. The imbalances influence disease-related factors and therefore provide some references for the prognosis and treatment of AL.

## 1. Introduction

Leukemia, a general term for malignant clonal disease of hematopoietic stem cells, is divided into myeloid and lymphoid according to cell types. Acute leukemia (AL) is the most common childhood hematological malignancy and is the leading cause of malignancy-related mortality in children [1]. Approximately 80% of children's AL cases are acute lymphoblastic leukemia (ALL) and 17% are acute myelogenous leukemia (AML) [2]. While a variety of factors have been suggested to be etiologically involved in leukemia, the etiology of leukemia is still unclear. Vitamins are essential nutrients for the human metabolism. As coenzymes or enzymes, vitamins play an important role in many important physiological processes, which contribute to normal body functions. In addition, vitamins have been reported to have preventive and therapeutic effects on some cancers [3, 4]. In children with AL, malnutrition is a common complication of the diseases and chemotherapy. Consequently, the resultant vitamins deficiency has been reported to negatively influence treatment response and disease prognosis [5]. It is reported that vitamin supplementation, particularly carotenoids and glutathione, may play a protective role against AL [3]. AL-caused oxidative stress response leads to increased concentration of vitamin C (VC) in leukocytes [4–6]. However, there are only a few studies on the effects of serum vitamin content on the pathogenesis or treatment of AL in children. Therefore, this study investigated the relationship between the serum vitamin content and disease-related indicators in children with AL.

## 2. Subjects and Methods

### 2.1. Study Subjects and Grouping

A total of 107 hospitalized children with AL (from June 2018 to December 2020) were enrolled in this study. The children were divided into the infected group (*n* = 52) and noninfected group (*n* = 55), according to the presence of infection. Bone marrow examination was conducted to evaluate remission and residual disease, and according to the examination results, the children were divided into the treatment remission group (no residual disease, *n* = 56) and nonremission group (with residual disease, *n* = 51). According to clinical risks and treatment responses, the children were divided into the high-risk (HR) group (*n* = 44), intermediate risk (IR) group (*n* = 53), and slight risk (SR) group (*n* = 8). According to different therapeutic regimens, the children were divided into three groups: cyclophosphamide + cytosine arabinoside + 6-mercaptopurine + pegaspargase group (CAML, *n* = 15), methotrexate group (MTX, *n* = 9), and vindesine + daunomycin + L-asparaginasum + prednisone (VALP, *n* = 38). Some other treatment groups (*n* = 45) were also set. The results in all the different groups were analyzed.

### 2.2. Methods

The fasting venous blood of all the study subjects was collected in the morning and stored at ambient temperatures for 1 h. Then, blood was centrifuged at 3000 rpm/min for 10 min. After that, serum was collected and stored in the fridge at −20°C. The serum vitamin content and blood-related disease indicators were determined using chemiluminescence with a vitamin detector (LK3000VI). Venous whole blood was collected for the routine blood analysis.

The disease-related indicators were as follows. (1) General information: age, body mass index (BMI), gender, diagnostic result type, immunophenotype, abnormal liver function, abnormal kidney function, and the occurrence of icterus. (2) Biochemical indicators: alanine aminotransferase (ALT), aspartate aminotransferase (AST), lactate dehydrogenase (LD), and hydroxybutyric dehydrogenase (HBDH). (3) Serological and hematological parameters: white blood count (WBC), neutrophils (N), lymphocyte (L), hemoglobin (Hb), platelet count (PLT), C-reactive protein (CRP), activated partial thromboplastin time (APTT), and troponin (Tn). (4) Vitamin (V) indicators: vitamin A (VA), VB1, VB2, VB6, VB9, VB12, VC, VD, and VE levels.

### 2.3. Statistical Methods

Statistical analysis was done using SPSS 21.0 software. Data were expressed as mean ± standard deviation (SD). If the data obeyed normal distribution and homogeneity of variance, the *t*-test or repeated measures analysis of variance was applied; otherwise, a nonparametric test was utilized. Multivariate analysis was performed using binary logistic regression. *P* < 0.05 was considered statistically significant.

## 3. Results

### 3.1. Analysis of Infection-Related Influencing Factors in Children with Acute Leukemia

The clinical general conditions of the children in infected and noninfected groups are given in Table 1. There were no significant differences in age, BMI, gender, diagnostic result type, immunophenotyping, abnormal liver and kidney function, and occurrence of icterus between the two groups (*P* > 0.05). LD and HBDH blood levels were significantly higher in the infected group than in the noninfected group (*P* < 0.05). Among the serological and hematological disease indicators, WBC, L, and CRP were significantly higher, while Hb and PLT were significantly lower in the infected group than in the noninfected group (*P* < 0.05). For various serum vitamins level, only VD was significantly lower in the infected group than that in the noninfected group (*P* < 0.05). Furthermore, multivariate regression analysis (Table 2) showed that Hb and CRP might be AL predisposing factors in children.

### 3.2. Analysis of Remission-Related Factors in Children with Acute Leukemia

Based on the disease status, the children were divided into the treatment remission group and nonremission group. There were no significant differences in age, BMI, gender, abnormal renal function, and occurrence of icterus between the two groups (*P* > 0.05). However, there were statistically significant differences in the diagnostic results, immunophenotype, liver function, and infection incidence (*P* < 0.05). The level of LD in the treatment remission group was significantly lower than that in the nonremission group (*P* < 0.05). Among the serological and hematological disease indicators, the levels of Hb, PLT, APTT, and Tn were significantly higher, while the levels of WBC and L were significantly lower in the treatment remission group than in the nonremission group (*P* < 0.05). For the serum vitamin levels, there was a statistically significant difference (*P* < 0.05) in VB1, VB6, and VB12 levels between the two groups (Table 3). Furthermore, the results of multivariate regression analysis showed that the type of leukemia (ALL or AML) may be a factor affecting AL remission in children (Table 4).

### 3.3. Analysis of Factors Influencing Different Risk Degrees in Children with Acute Leukemia

There were no significant differences in age, BMI, gender, diagnostic results, immunophenotype, and abnormal liver function among the general conditions (Table 5) among the HR, IR, and SR groups (*P* > 0.05). However, there were statistically significant differences in the occurrence of renal function and icterus (*P* < 0.05). There was a statistically significant difference in PLT among the three groups (*P* < 0.05). There were no statistically significant differences in serological and hematological parameters and vitamins levels (*P* < 0.05). The results of the multivariate regression analysis confirmed that abnormal renal function and icterus incidence were the influencing factors for risk degree in children with AL (Table 6).

### 3.4. Analysis of Treatment Regimen-Related Factors in Children with Acute Leukemia

There was no significant difference in age, BMI, gender, abnormal liver function, abnormal renal function, and icterus among the three therapeutic regimen groups (*P* < 0.05) (Table 7). However, there were statistically significant differences in immunophenotype and type of diagnosis (*P* < 0.05). For serological and hematological parameters, there were significant differences in N, PLT, and APTT among the three groups (*P* < 0.05). For serum vitamin levels, there was a statistically significant difference between VB6 and VB12 (*P* < 0.05). Furthermore, results from multivariate regression analysis showed that PLT was significantly higher and N was significantly lower in the CAML group than in the other regimen groups. The immunophenotype of the MTX group was statistically different from the other regimens. The VDLP group had lower APTT and higher VB6 compared to other regimens (*P* < 0.05). These results confirmed that PLT, N, immunophenotype, APTT, and VB6 were the factors that influenced the choice of AML treatment regimen in children (Table 8).

## 4. Discussion

In this study, a total of 107 AL children were included, and their vitamin content and clinical parameters were analyzed in relation to infection, disease status, and clinical risk and treatment regimens. According to the analysis results, the level of serum VD in the infected group was significantly lower than that in the noninfected group. Compared with the nonremission group, the serum levels of VB6 and VB12 in the treatment remission group were significantly decreased, while the level of VB1 was notably increased. Additionally, there were notable differences in the levels of VB6 and VB12 among treatment regimen groups.

Recently, it has been shown that vitamins have nonclassical effects such as regulating body immunity, inhibiting tumor cell proliferation, and participating in the development and progression of tumor cells [3, 4]. VD deficiency is a common malnutrition case. It affects approximately 30%–50% of the population worldwide, and most people are currently in a “subhealth” state of vitamin deficiency [7]. Relevant studies have shown that serum vitamins can affect peripheral blood T cells in children with pneumonia [8, 9]. Previous scholars have found that a decrease in VB6, VB9, and VB12 blood levels increases cancer risk, and epidemiological studies findings reported that adequate intake of folate, VB6, and VB12 may prevent breast cancer [10–12]. But the specific mechanism of action is not clear. However, these findings are not consistent with the results of this study. In our study, VB6 and VB12 serum levels were lower in the AL treatment remission group than in the nonremission group. Based on our analysis, since VB is involved in cell division as a coenzyme in the synthesis of purine and thymic acid for DNA synthesis [12], after treatment and remission of the patients, tumor cell division activity was reduced, so the level of VB6 and VB12 was significantly decreased in patients in the treatment remission group. Johansson et al. [13] measured the folic acid and VB12 blood concentrations in 869 patients and 1174 controls and concluded that VB12 may be associated with an increased risk of advanced prostate cancer. Chandy et al. [14] found that VB12 could increase colorectal cancer risk. Brasky et al. [15] demonstrated that the use of VB6 and VB12 alone without other vitamins increased the risk of lung cancer up to 30%–40% in men. In agreement with the present study, Pais et al. [16] showed that vitamin B6 levels were significantly higher in newly diagnosed childhood leukemia than in the control group. The possibility that folate has a dual regulatory effect depends on its timing and dose of administration. Folate supplementation before the onset of precancerous lesions may prevent tumor development, but increased folate in the presence of lesions may increase tumorigenesis [17, 18].

Giovannucci' study [19] showed that higher VD plays a protective role against the development of colorectal cancer and adenoma. There was a significant negative linear relationship between plasma VD and colorectal cancer risk [20]. Giovannucci et al. [21] showed that a 25 nmol/L increase in VD was associated with a 17% reduction in total cancer incidence, a 29% reduction in total cancer mortality, and a 43% and 45% reduction in digestive system cancer incidence and mortality, respectively. Together, the results of the above studies showed the protective effects of VD on tumorigenesis. In addition, a number of epidemiological studies were conducted in adults and children, and the results showed that VD deficiency was associated with an increased risk and severity of infections, especially respiratory infections [22]. Similarly, the results of this study also showed that VD levels were significantly lower in the infected group than in the noninfected group. Brasky et al. [15] also found that the level of VD in AL patients was significantly lower than the normal level.

PLT is the smallest cell fragment produced by megakaryocytes in the bone marrow. Under physiological conditions, PLT exerts the functions of adhesion, aggregation, release, and contraction to ensure smooth progress of the normal hemostatic process. PLT is also associated with pathological thrombosis, tumor metastasis, inflammation, and immune response [23]. AL is a common malignant proliferative tumor of the hematopoietic system. Bleeding is one of the common symptoms and causes of death in AL. The mechanism through which bleeding occurs is complex, involving various factors such as infiltration of leukemia cells into the vessel walls, the reduction of PLT production, and abnormal coagulation and anticoagulant functions. Among them, reduction of PLT production is the major cause of bleeding [24]. Studies have found that reduced PLT count in all types of AL may lead to abnormal PLT function [25, 26]. In this study, PLT count and Hb levels in the infected group were lower than those of in the noninfected group. The PLT count and Hb levels in the treatment remission group were significantly increased than those in the nonremission group. The PLT count also varied among the three risk degrees in children with AL. Together, these results indicate that low PLT count and Hb levels are associated with poor treatment outcomes and prognosis. Furthermore, the results of multivariate analysis showed that PLT was an influencing factor for the choice of AML treatment regimen.

CRP is commonly applied in the diagnosis of multiple systemic inflammatory diseases [27]. It has been reported that CRP can act as a marker of fever, bloodstream infection, and sepsis in immunocompromised patients [28–30]. Shimony et al. [31] demonstrated that CRP level was significantly elevated in AL, and as a sensitive biomarker, CRP preceded bloodstream infection. In this study, the level of CRP in the infected group was higher than that in the noninfected group. The level of CRP was lower in the treatment remission group than that in the nonremission group, but the differences were not significant. Multivariate analysis also confirmed that CRP level was a risk factor for the occurrence of infection in children with AL.

In this study, multivariate regression analysis results showed that abnormal renal function and icterus were effective prediction factors of different risk degrees in AL children, and L count, immunophenotype, and APTT were the influencing factors for the choice of therapeutic regimen. Overall, close attention to vitamin levels in AL children at different stages of chemotherapy, improvement of nutritional status, minimized complications, and especially reduction of the incidence of infection are important means to improve the survival rate and quality of life of AL children. However, due to the small sample size included in this study, some indicators had no significant changes at different stages of disease development in children with AL. Therefore, further studies with larger sample sizes are needed.

To sum up, this study has found imbalances in serum vitamins levels in AL children, which provide some references for AL diagnosis and treatment. The results of this study suggest that close attention to vitamins levels changes and maintaining vitamin level balance (through timely supplementation or cessation of vitamin intake) can contribute to successful treatment outcomes in children with AL. In addition, Hb and CRP were found to be the main factors influencing infection in children with AL. Since low HB is likely in AL patients, the risk of infections is high, and therefore, antiinfective treatment should be considered in the treatment of AL.

## Figures and Tables

**Table 1:** Analysis of infection-related influencing factors in children with acute leukemia.

Indicators		Infected group (*n* = 52)	Noninfected group (*n* = 55)	*t*/*X*^2^	*P* value

Age		7.54 ± 8.83	8.96 ± 16.95	0.901	0.370
BMI		16.88 ± 2.89	16.15 ± 2.76	1.335	0.100
Gender	Male	31 (59.6)	30 (54.5)	0.280	0.596
	Female	21 (40.4)	25 (45.5)		
Diagnostic results	ALL	42 (80.8)	42 (76.4)	0.307	0.579
	AML	10 (19.2)	13 (23.6)		
Immunophenotype	AML	9 (17.3)	13 (23.6)	3.028	0.220
	B	38 (73.1)	38 (69.1)		
	T	5 (9.6)	4 (7.3)		
Liver function (missing = 1)	Abnormal	17 (32.7)	12 (22.22)	1.461	0.227
	Normal	35 (67.3)	42 (77.78)		
Kidney function	Abnormal	12(23.1)	7 (12.7)	1.960	0.161
	Normal	40 (76.9)	48 (87.3)		
Icterus	Yes	2 (3.8)	6 (10.9)	1.928	0.165
	No	50 (96.2)	49 (89.1)		
Biochemical indicators	Alanine aminotransferase (ALT, mmol/L)	39.94 ± 92.14	38.38 ± 48.86	0.109	0.913
	Aspartate aminotransferase (AST, mmol/L)	39.02 ± 47.12	31.46 ± 23.50	1.049	0.297
	Lactate dehydrogenase (LD, U/L)	661.63 ± 1371.89	223.91 ± 65.42	2.364	**0.020** ^*∗*^
	Hydroxybutyric dehydrogenase (HBDH, U/L)	474.55 ± 906.57	168.80 ± 50.27	2.498	**0.014** ^*∗*^
Blood routine and serological parameters	White blood count (WBC, 10^9^/L)	14.99 ± 24.83	4.30 ± 4.53	3.139	**0.002** ^*∗*^
	Neutrophils (N, 10^9^/L)	3.66 ± 6.24	2.32 ± 2.19	1.489	0.140
	Hemoglobin (Hb, g/L)	80.17 ± 16.49	100.53 ± 20.85	5.581	**<0.001** ^*∗*^
	Platelet count (PLT, 10^9^/L)	108.46 ± 94.2	209.11 ± 112.59	5.000	**<0.001** ^*∗*^
	Lymphocyte (L, 10^9^/L)	7.57 ± 15.34	1.46 ± 2.16	2.928	**0.004** ^*∗*^
	C-reactive protein (CRP, mg/L)	13.87 ± 27.82	2.40 ± 8.59	2.361	**0.020** ^*∗*^
	Activated partial thromboplastin time (APTT, s)	29.22 ± 5.38	31.61 ± 7.16	1.930	0.056
	Troponin (Tn)	7.36 ± 9.68	6.49 ± 7.82	0.430	0.668
Vitamin level	Vitamin A (VA, *μ*mol/L)	0.73 ± 0.26	0.74 ± 0.18	0.400	0.690
	Vitamin B1 (VB1, nmol/L)	98.47 ± 11.71	100.05 ± 13.05	0.660	0.511
	Vitamin B2 (VB2, *μ*g/L)	5.45 ± 1.94	5.71 ± 1.75	0.732	0.466
	Vitamin B6 (VB6, nmol/L)	33.85 ± 14.54	33.80 ± 15.4	0.016	0.987
	Vitamin B9 (VB9, nmol/L)	20.19 ± 5.83	19.38 ± 5.76	0.723	0.471
	Vitamin B12 (VB12, pg/mL)	485.32 ± 102.97	472.17 ± 79.12	0.738	0.462
	Vitamin C (VC, *μ*mol/L)	39.22 ± 6.47	38.43 ± 4.54	0.728	0.469
	Vitamin D (VD, nmol/L)	37.96 ± 14.78	45.67 ± 19.97	2.259	**0.026** ^*∗*^
	Vitamin E (VE, *μ*g/mL)	10.76 ± 0.90	10.62 ± 0.56	0.956	0.341

Data were mean ± SD or *n* (%). ^*∗*^*P* < 0.05. AML, acute myeloid leukemia; BMI, body mass index.

**Table 2:** Multivariate regression analysis of influencing factors for infection in children with acute leukemia.

	B	Wald *X*^2^	Exp (B)	95% of Exp (B) confidence interval		*P*
				Lower limit	Upper limit	

Lactate dehydrogenase (LD)	0.002	0.022	1.002	0.975	1.031	0.881
Hydroxybutyric dehydrogenase (HBDH)	0.007	0.176	1.007	0.974	1.042	0.675
White blood cell count (WBC)	0.054	0.236	1.056	0.849	1.313	0.627
Hemoglobin (Hb)	−0.048	6.105	0.953	0.917	0.99	**0.013** ^*∗*^
Platelet count (PLT)	−0.002	0.215	0.998	0.992	1.005	0.643
Lymphocyte (L)	−0.009	0.004	0.991	0.76	1.292	0.949
C-reactive protein (CRP)	0.065	7.003	1.067	1.017	1.12	**0.008** ^*∗*^
Vitamin D (VD)	−0.039	3.35	0.961	0.922	1.003	0.067
Constant	3.205	4.53	24.654			0.033

^*∗*^ *P* < 0.05.

**Table 3:** Analysis of the factors influencing progression of acute leukemia in children.

Indicators		Treatment remission group (*n* = 56)	Nonremission group (*n* = 51)	*t*/*X*^2^	*P*

Age		6.32 ± 3.72	5.66 ± 3.40	0.955	0.342
BMI		16.02 ± 2.51	17.03 ± 3.09	1.848	0.060
Gender	Male	31 (55.4)	30 (58.8)	0.131	0.718
	Female	25 (44.6)	21 (41.2)		
Diagnostic results	ALL	49 (87.5)	35 (68.6)	5.966	**0.010** ^*∗*^
	AML	7 (12.5)	16 (31.4)		
Immunophenotype	AML	7 (12.5)	15 (29.4)	6.309	**0.043** ^*∗*^
	B	42 (75.0)	34 (66.7)		
	T	7 (12.5)	2 (3.9)		
Liver function	Abnormal	20 (36.4)	9 (17.6)	4.664	**0.030** ^*∗*^
Kidney function	Normal	36 (63.6)	42 (82.4)		
Icterus	Abnormal	13 (23.2)	6 (11.8)	2.396	0.122
	Normal	43 (76.8)	45 (88.2)		
Liver function (missing = 1)	Yes	4 (7.1)	4 (7.8)	0.019	0.890
	No	52 (92.9)	47 (92.2)		
Infection	Yes	18 (32.1)	34 (66.7)	12.735	**<0.001** ^*∗*^
	No	38 (67.9)	17 (33.3)		
Biochemical indicators	Alanine aminotransferase (ALT, mmol/L)	42.93 ± 51.65	34.24 ± 90.83	0.610	0.543
	Aspartate aminotransferase (AST, mmol/L)	39.93 ± 40.17	29.50 ± 32.30	1.457	0.148
	Lactate dehydrogenase (LD, U/L)	231.11 ± 80.66	656.14 ± 1373.01	2.207	**0.032** ^*∗*^
	Hydroxybutyric dehydrogenase (HBDH, U/L)	170.00 ± 59.74	475.02 ± 906.01	2.399	0.200
Serological indicators	White blood cell count (WBC, 10^9^/L)	4.16 ± 3.50	15.34 ± 25.14	3.149	**0.003** ^*∗*^
	Neutrophils (N, 10^9^/L)	2.73 ± 2.50	3.24 ± 6.24	0.547	0.587
	Hemoglobin (Hb, g/L)	99.79 ± 20.05	80.59 ± 18.14	5.175	<**0.001**^*∗*^
	Platelet count (PLT)	183.00 ± 102.30	135.16 ± 124.19	2.182	**0.031** ^*∗*^
(PLT, 10^9^/L)	Lymphocyte (L, 10^9^/L	1.05 ± 1.16	8.14 ± 15.39	3.286	**0.002** ^*∗*^
	C-reactive protein (CRP, mg/L)	7.14 ± 15.54	8.89 ± 25.93	0.426	0.671
	Activated partial thromboplastin time (APTT, s)	32.76 ± 7.29	28.03 ± 4.24	4.118	<**0.001**^*∗*^
	Troponin (Tn)	9.24 ± 10.03	5.20 ± 5.33	2.533	**0.01** ^*∗*^
Vitamin level	Vitamin A (VA, *μ*mol/L)	0.74 ± 0.18	0.73 ± 0.26	0.141	0.888
	Vitamin B1 (VB1, nmol/L)	102.58 ± 12.53	95.67 ± 11.27	3.003	**0.003** ^*∗*^
	Vitamin B2 (VB2, *μ*g/L)	5.72 ± 1.81	5.44 ± 1.88	0.793	0.430
	Vitamin B6 (VB6, nmol/L	30.41 ± 13.29	37.58 ± 15.81	2.547	**0.012** ^*∗*^
	Vitamin B9 (VB9, nmol/L	20.55 ± 5.78	18.92 ± 5.71	1.468	0.145
	Vitamin B12 (VB12, pg/mL	453.54 ± 73.62	506.03 ± 101.17	3.043	**0.003** ^*∗*^
	Vitamin C (VC, *μ*mol/L	39.57 ± 5.77	37.99 ± 5.23	1.482	0.141
	Vitamin D (VD, nmol/L	44.93 ± 20.64	38.63 ± 13.98	1.828	0.070
	Vitamin E (VE, *μ*g/mL)	10.69 ± 0.75	10.70 ± 0.75	0.057	0.955

Data were mean ± SD or *n* (%). ^*∗*^*P* < 0.05. AML, acute myeloid leukemia; BMI, body mass index.

**Table 4:** Multivariate regression analysis of factors affecting remission in children with acute leukemia.

	B	Standard error	Wald *X*^2^	*P*	Exp (B)

Diagnostic results	2.372	0.924	6.596	**0.01**	10.724
Abnormal liver function	0.395	1.065	0.137	0.711	1.484
Infection	1.501	1.032	2.117	0.146	4.486
Lactate dehydrogenase (LD)	0	0	0.056	0.813	1
White blood cell count (WBC)	0.029	0.026	1.291	0.256	1.03
Hemoglobin (Hb)	0.027	0.026	1.059	0.304	1.028
Platelet count (PLT)	−0.001	0.005	0.035	0.851	0.999
Lymphocyte (L)	−0.033	0.052	0.394	0.53	0.968
Activated partial thromboplastin time (APTT)	−0.009	0.074	0.015	0.904	0.991
Troponin (Tn)	−0.043	0.037	1.389	0.239	0.958
Vitamin B1 (VB1)	−0.012	0.035	0.129	0.719	0.988
Vitamin B6 (VB6)	0.001	0.033	0.002	0.968	1.001
Vitamin B12 (VB12)	−0.011	0.006	3.777	0.052	0.989
Constant	3.355	4.885	0.472	0.492	28.655

The value with P > 0.05 is indicated in bold.

**Table 5:** Analysis of factors influencing different risk degrees in children with acute leukemia.

Indicators		HR group (*n* = 44)	IR group (*n* = 53)	SR group (*n* = 8)	*F*/*X*^2^	*P*

Age		8.18 ± 10.83	8.98 ± 16.57	5.25 ± 2.92	0.261	0.771
BMI		16.85 ± 2.78	16.58 ± 2.88	14.43 ± 2.5	0.883	0.417
Gender	Male	22 (50)	33 (62.3)	4 (50.0)	1.604	0.448
	Female	22 (50)	20 (37.7)	4 (50.0)		
Diagnostic results	ALL	35 (79.5)	40 (75.5)	7 (87.5)	0.681	0.711
	AML	9 (20.5)	13 (24.5)	1 (12.5)		
Immunophenotype	AML	8 (18.2)	13 (24.5)	1 (12.5)	1.084	0.897
	B	32 (72.7)	36 (67.9)	6 (75.0)		
	T	4 (9.1)	4 (7.5)	1 (12.5)		
Liver function	Abnormal	10 (22.7)	16 (30.8)	1 (12.5)	2.119	0.347
	Normal	34 (77.3)	36 (69.2)	7 (87.5)		
Renal function	Abnormal	4 (9.1)	11 (20.8)	4 (50.0)	9.869	**0.007** ^*∗*^
	Normal	40 (90.9)	42 (79.2)	4 (50.0)		
Icterus	Yes	5 (11.4)	8 (15.1)	0	8.496	**0.014** ^*∗*^
	No	39 (88.6)	45 (84.9)	8 (100.0)		
Biochemical indicator	Alanine aminotransferase (ALT, mmol/L)	48.11 ± 106.33	31.58 ± 34.05	47.49 ± 36.33	0.641	0.529
	Aspartate aminotransferase (AST, mmol/L)	41.51 ± 50.47	29.78 ± 23.77	39.57 ± 17.33	1.230	0.297
	Lactate dehydrogenase (LD, U/L)	534.66 ± 1281.05	363.04 ± 728.54	303.86 ± 181.69	0.426	0.654
	Hydroxybutyric dehydrogenase (HBDH, U/L)	386.91 ± 841.45	262.06 ± 491.06	239.14 ± 161.26	0.487	0.616
Serological indicators	White blood cell count (WBC, 10^9^/L)	6.99 ± 11.62	12.37 ± 23.50	5.83 ± 4.62	1.203	0.304
	Neutrophils (N, 10^9^/L)	3.33 ± 5.50	2.80 ± 4.29	2.72 ± 1.66	0.168	0.846
	Hemoglobin (Hb, g/L)	87.89 ± 18.32	92.45 ± 22.68	97.88 ± 28.54	0.997	0.373
	Platelet count (PLT)	125.39 ± 87.45	189.85 ± 132.01	170.63 ± 92.35	3.964	**0.022** ^*∗*^
(PLT, 10^9^/L)	Lymphocyte (L, 10^9^/L)	2.76 ± 6.16	6.18 ± 14.67	2.63 ± 3.98	1.224	0.298
	C-reactive protein (CRP, mg/L)	9.63 ± 25.49	9.15 ± 19.36	9.21 ± 14.44	0.006	0.994
	Activated partial thromboplastin time (APTT, s)	30.73 ± 7.70	30.61 ± 5.76	28.36 ± 2.57	0.411	0.664
	Troponin (Tn)	6.79 ± 8.58	5.68 ± 8.62	6.28 ± 11.67	0.192	0.826
Vitamin level	Vitamin A (VA, *μ*mol/L)	0.71 ± 0.18	0.76 ± 0.24	0.71 ± .24	0.944	0.392
	Vitamin B1 (VB1, nmol/L)	98.32 ± 13.29	99.91 ± 12.16	101.67 ± 10.33	0.336	0.715
	Vitamin B2 (VB2, *μ*g/L)	5.42 ± 1.33	5.78 ± 2.25	5.50 ± 1.37	0.466	0.629
	Vitamin B6 (VB6, nmol/L)	34.77 ± 17.05	32.86 ± 13.23	36.43 ± 15.96	0.309	0.735
	Vitamin B9 (VB9, nmol/L)	20.49 ± 6.73	19.54 ± 5.04	18.14 ± 4.94	0.688	0.505
	Vitamin B12 (VB12, pg/mL)	484.54 ± 91.76	474.32 ± 90.16	446.55 ± 76.09	0.635	0.532
	Vitamin C (VC, *μ*mol/L)	38.69 ± 5.26	39.22 ± 6.10	37.51 ± 3.45	0.358	0.700
	Vitamin D (VD, nmol/L)	40.85 ± 15.11	44.04 ± 21.09	36.56 ± .02	0.785	0.459
	Vitamin E (VE, *μ*g/mL)	10.77 ± 0.83	10.62 ± 0.68	10.77 ± 0.87	0.520	0.596

Data were mean ± SD or *n* (%). Missing = 2. ^*∗*^*P* < 0.05. AML, acute myeloid leukemia; BMI, body mass index; HR, high risk; IR, intermediate risk; SR, slight risk.

**Table 6:** Multivariate regression analysis of factors influencing different risk degrees in children with acute leukemia.

Slight risk (SR = 0)		B	Wald *X*^2^	Exp (B)	95% of Exp (B) confidence interval		*P*
					Lower limit	Upper limit	

HR	Platelet count (PLT, 10^9^/L)	−0.006	0.004	0.997	0.987	1.002	0.167
	Abnormal renal function = 1.00	−2.558	7.247	0.077	**0.012**	**0.499**	**0.007** ^*∗*^
	Icterus = 1.00	19.288	372.102	237982258.740	33530638.034	1689068827.669	<**0.001**^*∗*^
	Constant	2.968					

IR	Platelet count (PLT, 10^9^/L)	0.001	0.103	1.001	0.994	1.008	0.749
	Abnormal renal function = 1.00	−1.356	2.970	0.258	0.055	1.205	0.085
	Icterus = 1.00	17.149	0.000	28035276.423	28035276.422843	28035276.423	<**0.001**^*∗*^
	Constant	2.106					

^*∗*^ *P* < 0.05. HR, high risk; IR, intermediate risk; SR, slight risk.

**Table 7:** Analysis of factors influencing different treatment regimens in children with acute leukemia.

Indicators		CAML group (*n* = 15)	MTX group (*n* = 9)	VDLP group (*n* = 38)	Other groups (*n* = 45)	F/*X*^2^	*P*

Age		6.22 ± 4.46	4.93 ± 2.67	5.18 ± 2.95	6.92 ± 3.63	2.483	0.065
BMI		16.54 ± 3.28	16.24 ± 2.51	16.59 ± 2.90	16.45 ± 2.77	0.043	0.988
Gender	Male	7 (46.67)	4 (44.44)	23 (60.53)	27 (60.00)	1.590	0.662
	Female	8 (53.33)	5 (55.55)	15 (39.47)	18 (40.00)		
Diagnostic results	AML	0	1 (11.11)	0	22 (48.89)	35.098	<**0.001**^*∗*^
	ALL	15 (100.00)	8 (88.89)	38 (100.0)	23 (51.11)		
Immunophenotype	B	15 (100.00)	5 (55.55)	37 (97.37)	19 (42.22)	47.056	<**0.001**^*∗*^
	T	0	3 (33.33)	1 (2.63)	5 (11.11)		
	AML	0	1 (11.11)	0 (2.9)	21 (46.67)		
Liver function	Abnormal	2 (26.67)	3 (33.33)	9 (23.68)	15 (33.33)	2.908	0.406
	Normal	13 (73.33)	6 (66.67)	29 (76.32)	29 (64.44)		
Renal function	Abnormal	6 (40.00)	2 (22.22)	6 (15.79)	5 (11.11)	6.666	0.083
	Normal	9 (60.0)	7 (77.78)	32 (84.21)	40 (88.89)		
Icterus	Yes	1 (6.67)	1 (11.11)	1 (2.63)	5 (11.11)	2.335	0.506
	No	14 (93.33)	8 (88.89)	37 (97.37)	40 (88.89)		
Biochemical indicator	Alanine aminotransferase (ALT, mmol/L)	20.68 ± 14.95	40.89 ± 23.79	47.79 ± 104.97	37.56 ± 55.13	0.502	0.682
	Aspartate aminotransferase (AST, mmol/L)	22.66 ± 5.71	37.66 ± 14.25	33.11 ± 39.72	40.75 ± 42.94	0.953	0.418
	Lactate dehydrogenase (LD, U/L)	215.33 ± 44.06	235.67 ± 41.50	374.24 ± 307.76	601.95 ± 1473.89	0.858	0.465
	Hydroxybutyric dehydrogenase (HBDH, U/L	164.67 ± 36.99	2.36 ± 3.30	293.61 ± 223.21	414.68 ± 974.95	0.763	0.517
Serological indicators	White blood cell count (WBC, 10^9^/L)	2.27 ± 1.75	4.32 ± 1.33	10.30 ± 18.23	12.25 ± 22.29	1.394	0.249
	Neutrophils (N, 10^9^/L)	1.46 ± 1.22	3.22 ± 1.61	1.57 ± 1.74	4.61 ± 6.59	3.846	**0.012** ^*∗*^
	Hemoglobin (Hb, g/L)	9.09 ± 1.67	98.56 ± 16.30	84.68 ± 20.73	94.00 ± 23.38	1.807	0.151
	Platelet (PLT, 10^9^/L	2.26 ± 1.09	171.11 ± 88.49	171.00 ± 133.53	126.84 ± 94.98	3.233	**0.025** ^*∗*^
	Lymphocyte (L, 10^9^/L)	0.62 ± 0.46	0.85 ± 0.42	7.53 ± 14.78	3.80 ± 10.06	1.961	0.124
	C-reactive protein (CRP, mg/L)	7.67 ± 17.66	5.60 ± 11.21	6.99 ± 26.19	10.43 ± 20.52	0.225	0.879
	Activated partial thromboplastin time (APTT, s)	35.31 ± 9.31	31.26 ± 4.89	26.63 ± 3.54	31.96 ± 5.88	10.267	<**0.001**^*∗*^
	Troponin (Tn)	8.92 ± 4.17	13.88 ± 13.80	5.02 ± 2.91	10.43 ± 10.97	1.370	**0.261**
Vitamin level	Vitamin A (VA, *μ*mol/L)	0.81 ± 0.20	0.79 ± 0.16	0.70 ± 0.27	0.73 ± 0.18	1.173	0.324
	Vitamin B1 (VB1, nmol/L)	101.03 ± 13.23	100.91 ± 14.64	95.16 ± 11.22	101.85 ± 12.08	2.279	0.084
	Vitamin B2 (VB2, *μ*g/L)	5.29 ± 0.88	4.73 ± 0.66	5.53 ± 1.68	5.90 ± 2.28	1.247	0.297
	Vitamin B6 (VB6, nmol/L)	32.83 ± 13.74	29.82 ± 12.24	40.03 ± 16.67	29.72 ± 12.68	3.854	**0.012** ^*∗*^
	Vitamin B9 (VB9, nmol/L)	2.06 ± 5.36	21.76 ± 7.45	18.53 ± 5.28	20.14 ± 5.93	1.113	0.347
	Vitamin B12 (VB12, pg/mL)	434.05 ± 54.62	435.39 ± 74.77	515.39 ± 98.76	470.93 ± 87.31	4.415	**0.006** ^*∗*^
	Vitamin C (VC, *μ*mol/L)	40.16 ± 7.20	39.71 ± 3.98	38.25 ± 5.80	38.67 ± 5.04	0.507	0.204
	Vitamin D (VD, nmol/L)	50.22 ± 23.74	39.16 ± 10.24	37.98 ± 13.87	43.05 ± 19.46	1.954	0.678
	Vitamin E (VE, *μ*g/mL)	10.49 ± 0.48	10.60 ± 0.59	10.78 ± 0.86	10.70 ± 0.75	1.846	0.144

Data were mean ± SD or *n* (%). Missing = 13. AML, acute myeloid leukemia; BMI, body mass index; CAML, cyclophosphamide + cytosine arabinoside+6-mercaptopurine + pegaspargase; MTX, methotrexate; VDLP, vindesine + daunomycin + L-asparaginasum + prednisone. The value with P > 0.05 is indicated in bold.

**Table 8:** Multivariate analysis of factors influencing different treatment regimens in children with acute leukemia.

Regimen (others = 0)		B	Wald *X*^2^	Exp (B)	95% of Exp (B) confidence interval		*P*
					Lower limit	Upper limit	

CAML	Intercept	0.548	0				1
	Platelet count (PLT)	0.01	4.682	1.01	1.001	1.019	**0.030** ^*∗*^
	Neutrophils (N)	−0.801	4.969	0.449	0.222	0.908	**0.026** ^*∗*^
	Activated partial thromboplastin time (APTT)	0.022	0.148	1.022	0.915	1.141	0.701
	Vitamin B6 (VB6)	−0.013	0.177	0.987	0.927	1.05	0.674
	Vitamin B12 (VB12)	−0.003	0.471	0.997	0.987	1.006	0.492
	Immunophenotype = 0.00^a^	0.165	0	1.18*E* + 00	0		1.00*E* + 00
	Immunophenotype = 1.00^b^	−17.98	0	1.55*E* − 08	0		9.99*E* − 01
	Diagnosis = 0^c^	−17.335	0	2.96*E* − 08	0		0.999

MTX	Intercept	19.84	20.885				0
	Platelet count (PLT)	0.002	0.369	1.002	0.995	1.01	0.543
	Neutrophils (N)	0.005	0.002	1.005	0.799	1.264	0.968
	Activated partial thromboplastin time (APTT)	−0.078	0.86	0.925	0.784	1.091	0.354
	Vitamin B6 (VB6)	−0.016	0.23	0.984	0.921	1.052	0.632
	Vitamin B12 (VB12)	−0.005	0.849	0.995	0.984	1.006	0.357
	Immunophenotype = 0.00^a^	−16.297	177.051	8.37*E* − 08	7.59*E* − 09	9.23*E* − 07	<**0.001**^*∗*^
	Immunophenotype = 1.00^b^	−15.147	125.811	2.64*E* − 07	1.87*E* − 08	3.73*E* − 06	<**0.001**^*∗*^
	Diagnosis = 0^c^	−17.91	.	1.67*E* − 08	1.67*E* − 08	1.67*E* − 08	.

VDLP	Intercept	10.317	0				0.999
	Platelet count (PLT)	0.001	0.143	1.001	0.994	1.008	0.705
	Neutrophils (N)	−0.499	5.798	0.607	0.405	0.911	**0.016** ^*∗*^
	Activated partial thromboplastin time (APTT)	−0.412	10.908	0.662	0.518	0.846	**0.001** ^*∗*^
	VB6	0.065	4.721	1.067	1.006	1.131	**0.030** ^*∗*^
	VB12	0.007	2.348	1.007	0.998	1.016	0.125
	Immunophenotype = 0.00^a^	−2.274	0	0.103	0	.b	1
	Immunophenotype = 1.00^b^	−3.488	0	0.031	0	.b	1
	Diagnosis = 0^c^	−20.163	0	1.75*E* − 09	0	.b	0.998

^*∗*^ *P* < 0.05. ^a^AML was considered as the control group of immunophenotype, B cell type: immunophenotype = 0.00; ^b^T cell type: immunophenotype = 1.00; ^c^ALL acted as the control group of diagnostic results, AML: diagnosis = 0. CAML, cyclophosphamide + cytosine arabinoside+6-mercaptopurine + pegaspargase; MTX, methotrexate group; VDLP, vindesine + daunomycin + L-asparaginasum + prednisone.

## Data Availability

The data used to support the findings of this study are available from the corresponding author upon request.
